The article "Cedrus deodara: In Vivo Investigation of Burn Wound Healing Properties" was published in 2023. Journal: Evid Based Complement Alternat Med.

# *Cedrus deodara: In Vivo* Investigation of Burn Wound Healing Properties

**DOI:** 10.1155/2023/5596964

**Published:** 2023-04-07

**Authors:** Arezoo Rastegari, Azadeh Manayi, Tahmineh Akbarzadeh, Reza Hojjatifard, Nasrin Samadi, Mahnaz Khanavi, Somayeh Niknam, Mina Saeedi

**Affiliations:** ^1^Persian Medicine and Pharmacy Research Center, Tehran University of Medical Sciences, Tehran, Iran; ^2^Medicinal Plants Research Center, Faculty of Pharmacy, Tehran University of Medical Sciences, Tehran, Iran; ^3^Department of Medicinal Chemistry, Faculty of Pharmacy, Tehran University of Medical Sciences, Tehran, Iran; ^4^Department of Pharmacognosy, Faculty of Pharmacy, Tehran University of Medical Sciences, Tehran, Iran; ^5^Department of Drug and Food Control, Faculty of Pharmacy and Pharmaceutical Quality Assurance Research Center, Tehran University of Medical Sciences, Tehran, Iran; ^6^Faculty of Land and Food Systems, University of British Columbia, Vancouver, British Columbia V6T 1Z4, Canada; ^7^Department of Pharmaceutics, Faculty of Pharmacy, Tehran University of Medical Sciences, Tehran, Iran

## Abstract

**Objective:**

*Cedrus deodara* (Roxb. Ex Lamb.) G. Don possesses various biological activities, which have been documented in modern and traditional medicine. In this study, burn wound healing activity of the methanol extract of* C. deodara* wood was evaluated *via* a burn wound model in Wistar rats.

**Methods:**

The methanol extract of *C. deodara* was evaluated for the contents of phenolic compounds, flavonoids, and tannins. Also, its antioxidant activity was determined using the DPPH assay. Then, a topical ointment containing the methanol extract of *C. deodara* (10%) was used to evaluate the healing effects on a model of second-degree thermal burn in 4 groups of 7 rats within 21 days. In this respect, average wound surface area, wound closure, and various histological features were examined.

**Results:**

Our findings revealed that the wounds treated with the methanol extract of *C. deodara* showed higher wound contraction (33.6, 87.1, and 93.4% on days 7, 14, and 21, respectively) compared with the positive control (27.6, 80.7, and 88.3% on days 7, 14, and 21, respectively) and the negative control (20.1, 77.9, and 80.2% on days 7, 14, and 21, respectively). According to the results from epitheliogenesis score, the number of inflammatory cells, neovascularization, and collagen density, good burn wound healing activity of the methanol extract of *C. deodara*was demonstrated.

**Conclusion:**

Using the methanol extract of *C. deodara* in an ointment formulation can be developed to prevent or reduce burn injury progression.

## 1. Introduction

Burns are skin injuries usually caused by excessive heat, electricity, radioactivity, or corrosive chemicals, which need careful monitoring at each step of healing. They have been a global public issue, leading to an estimated 180,000 deaths annually. The destructive outcomes of burns include physical disabilities as well as mental and emotional disorders, which impose high costs on societies [1]. Burn wound healing is a complex process consisting of several phases: inflammation, re-epithelialization, granulation tissue formation, and remodeling of extracellular matrix. Infections have been found as one of the main concerns delaying wound healing process and despite the discovery of a vast spectrum of antiseptics, it still remains a challenge to modern medicine [2]. Adverse effects of topical antibacterial agents and disinfectants include allergic reactions, skin irritations as well as the possibility of antimicrobial resistance, which can reduce the rate of skin repair and increase the rehabilitation period [3].

Natural products have shown promising properties in the wound healing process through different mechanisms of action [4]. Extracts [5–8], essential oils [9, 10], and secondary metabolites [11] isolated from medicinal plants were found to be effective.

*Cedrus deodara* (Roxb. ex Lamb.) G. Don., commonly known as deodar, is a species of western Himalayan cypress tree belonging to the Pinaceae family. It locally grows in eastern Afghanistan, northern Pakistan, northwestern India, southwestern Tibet, and western Nepal [12]. Different parts of the plant have been traditionally used for the treatment of various diseases such as arthritis, asthma, gastric disturbances, inflammation, microbial infections, and neurological and skin disorders. The leaf and resin paste of the plant has been topically used for wound healing [13]. Phytochemistry studies of *C. deodara* extracts and oils have indicated more than one hundred constituents including flavonoids, lignans, sterols, terpenoids, terpenes, sesquiterpene, and hydrocarbons [13]. In this work, burn wound healing of the methanol extract of *C. deodara* wood was evaluated in a topical formulation (ointment) *via* an *in vivo* burn model.

## 2. Materials and Methods

All solvents and reagents were obtained from Merck and Aldrich. *S. aureus* ATCC 6538 and *P. aeruginosa* ATCC 9027 were provided by the Iranian Research Organization for Science and Technology (IROST). Xylazine, ketamine, silver sulfadiazine (1%) ointment, and eucerin 400 were obtained from the pharmacy of Imam Khomeini Hospital Complex.

### 2.1. Plant Material

Four- to five-year-old branches of *Cedrus deodara* (Roxb. ex Lamb.) G. Don. (Figure 1) were obtained from the Nowshahr Botanical Garden, Iran. They were identified and voucher specimen of 7079-TEH was deposited in the Herbarium of the Faculty of Pharmacy, Tehran University of Medical Sciences, Tehran, Iran.

### 2.2. Preparation of the Methanol Extract

Dried branches of *C. deodara *(1000 g) were cut and powdered. The methanol (80%) extract was prepared by maceration of powder in three 72 h rounds at room temperature. The extract was concentrated under vacuum (Heidolph, Heizbad Hei-VAP, Germany) at 25°C and then lyophilized by a laboratory freeze dryer (LTE Science LTD, England) to obtain a dry and brittle powder (137 g).

### 2.3. Phytochemical Analysis

The methanol extract of *C. deodara* was phytochemically analyzed by measurement of the total phenolic, flavonoid, and tannin contents. Also, the antioxidant activity of the extract was evaluated by DPPH radical scavenging assay.

### 2.4. Determination of Total Phenolic Content

The total phenolic content was determined using the Folin–Ciocalteu reagent and expressed as gallic acid equivalent [14].

### 2.5. Determination of Total Flavonoid Content

Total flavonoid content was measured using the aluminum chloride method and expressed in terms of catechin equivalent, based on the described method in our previous work [15].

### 2.6. Determination of Total Tannin Content

Total tannin content was determined as described in the literature and expressed as tannic acid equivalent [16].

### 2.7. DPPH Radical Scavenging Activity

The antioxidant activity of the extract was evaluated using DPPH (1,1-diphenyl-2-picrylhydrazyl), compared with butylated hydroxyanisole (BHA), according to the literature [14].

### 2.8. Antimicrobial Assay

Minimum inhibitory concentrations (MICs) of the methanol extract of *C. deodara* were determined by agar dilution method against *Staphylococcus aureus* ATCC 6538 as a Gram-positive and *Pseudomonas aeruginosa* ATCC 9027 as a Gram-negative bacterium. Two-fold dilutions of the extract were prepared in dimethyl sulfoxide (DMSO). Each dilute was added to molten Mueller–Hinton (MH) agar (1 : 19 mL) at 50°C to give the final concentrations of 20, 10, 5, 2.5, 1.25, 0.63, and 0.31 mg/mL. The plates were spot inoculated with 3 *μ*L of each bacterial suspension in sterile saline (10^4^ CFU/spot), including a control plate containing 1 mL DMSO. The plates were incubated at 37°C for 24 h. Ciprofloxacin was used as the positive control in a side-by-side comparison with test antimicrobial agent. The MIC was determined as the lowest concentration of the agent that completely inhibits visible growth of the microorganisms [17].

### 2.9. Burn Wound Healing Activity of *C. deodara*

The study was approved by the Committee of Ethics of the Faculty of Pharmacy of Tehran University of Medical Sciences with approval number: IR.TUMS.VCR.REC.1398.584.

### 2.10. Experimental Animals

Twenty-eight Wistar male rats (200–220 g) of approximately eight weeks of age were studied and randomly divided into four groups of seven rats. The animals were housed in the standard environmental conditions (temperature: 22 ± 3°C, humidity: 60 ± 5%, and a 12 h light/dark cycle). During the experiment, the rats were fed a standard pellet diet (Pastor Institute, Iran) and water *ad libitum*. All procedures were carried out according to the institutional guidelines for animal care and use.

### 2.11. Preparation of Ointment

The topical ointment formulation (10%) was accordingly prepared: 20 g of the methanol extract of *C. deodara* was dissolved in 20 mL distilled water, and eucerin 400% was gradually added to the resulting solution to obtain 200 g of ointment, which was then well mixed to afford a homogenous product (final concentration of extract: 10%). Also, an ointment base (eucerin 400%) with no extract was used as a placebo (negative control).

### 2.12. Burn Wound Model

A burn wound model was used to evaluate the healing activity of the methanol extract of *C. deodara*. After inducing anesthesia *via* the intraperitoneal injection of 2% xylazine (5 mg/kg) and 10% ketamine (100 mg/kg), the rats were fixed in a ventral posture on a surgery table. The hair on the backs of the rats was covered in shaving cream and washed off after 10 minutes, so that no wounds were created in these areas. Deep second-degree burns were created by a circular probe with a diameter of 1.5 cm using a standard burn device (110°C for 10 seconds). Burn wounds were washed with physiological saline.

### 2.13. Grouping Animals

The animals were numbered, weighed, and randomly divided into four groups of seven rats:

*O* group: rats treated with ointment base with no extract as placebo (negative control).

*P* group: rats treated with a topical ointment containing 10% (w/w) of the methanol extract of *C. deodara*.

NC group: rats treated with nothing and only dressed in sterile gauze to assess “normal” wound healing (Normal healing group).

PC group: rats treated with “silver sulfadiazine (1%) ointment” as the positive control.

After creating burns on the rats' backs, all groups were first treated with only sterile gauze for 24 h to allow the wounds to expand. Then, topical ointments (extract and placebo) were applied to the wound surface using sterile gauze. For the positive control group (PC), the ointment was also applied to the wound using sterile gauze. The dressings were changed every 24 h. All rats were monitored daily for 21 days. Wound size was calculated using Adobe Photoshop CC 2018 (Adobe Systems Inc.).

### 2.14. Statistical Analysis

For the parametric data, the difference between groups were evaluated by one-way analysis of variance (ANOVA) followed by Tukey's post hoc test for multiple comparisons. *P* values less than 0.05 were considered significant.

### 2.15. Histopathological Studies

Animals from each group were euthanized at 7-, 14-, and 21-days postinjury (DPI), and the skin tissues were harvested and immediately fixed in the 10% neutral buffered formalin (pH = 7.26) for 48 h. The fixed tissue samples were then processed, embedded in paraffin, and sectioned to 5 *μ*m thickness. Finally, the sections were stained with haematoxylin and eosin (H&E). The histological slides were evaluated by two independent reviewers, using light microscopy (Olympus BX51; Olympus, Tokyo, Japan) in a double-blind fashion. Angiogenesis, inflammatory cell infiltration, and fibroplasia (collagen content) were assessed in different groups, comparatively. Magnification × 400 was employed to count different cells and calculations were repeated in five fields. Finally, the average number of each criterion for these fields was recorded. Epithelialization was assessed at 7, 14 and 21 DPI, semiquantitatively on 5-point scores: 0 (without new epithelialization), 1 (25%), 2 (50%), 3 (75%), and 4 (100%) epithelialization. For these parameters, the results were validated by a comparative analysis of two independent observers blinded to the treatment groups.

### 2.16. Statistical Analysis

For parametric data, the difference between groups were evaluated by one-way analysis of variance (ANOVA) followed by Tukey's post hoc test for multiple comparisons. *P* values less than 0.05 were considered significant.

## 3. Results

### 3.1. Extraction Yield and Phytochemical Analysis

The yield of methanol extract of *C. deodara* was calculated as 13.7%. Also, the total phenolic, flavonoid, and tannin contents were assayed as reported in Table 1.

### 3.2. 1,1-Diphenyl-2-picrylhydrazyl (DPPH) Radical Scavenging Activity

The methanol extract of *C. deodara* was investigated for its DPPH radical scavenging activity in comparison to BHA as the reference antioxidant agent (IC_50_ = 91.28 ± 0.13 *μ*g/mL). It depicted very good antioxidant activity with IC_50_ value of 10.6 ± 0.80 *μ*g/mL.

### 3.3. Antibacterial Assay

Antibacterial activity of the methanol extract of *C. deodara* was evaluated against two Gram-positive and Gram-negative strains, *Staphylococcus aureus* and *Pseudomonas aeruginosa*, respectively (Table 2). It showed pronounced antibacterial activity against *S. aureus*.

### 3.4. Burn Wound Healing Activity of *C. deodara*

The wound area was measured on the 0, 1st, 7th, 14th, and 21st days after burn in all groups using Adobe Photoshop CC 2017. Wound surface reduction was recorded in Table 3. The percentage of wound contraction (wound closure) was also calculated according to equation (1) (Table 4).

(1) $$\begin{array}{c} Wound\;closure\;\left(\%\right)=\left[\frac{\left(wound\;surface\;area\;on\;day\;n-wound\;surface\;area\;on\;day\;1\right)}{wound\;surface\;area\;on\;day\;1}\right]*100\text{.} \end{array}$$

As shown in Table 3, group P containing the methanol extract of *C. deodara* showed remarkable decrease in wound surface area compared with groups O, NC, and PC especially at 21-day postinjury.

According to Table 4, the percentage of wound closure within 21 days was significantly increased for group *P* compared with the other groups (*P* < 0.05). On both days 14 and 21, group P demonstrated significantly higher wound contraction compared to groups O, NC, and PC (*P* < 0.001, *P* ≤ 0.001, and *P* < 0.05, respectively).

### 3.5. Histopathological Studies

All groups were studied for histopathological changes using light microscopy as shown in Figure 2. The histopathologic evaluation of lesions in the NC group showed the granulation tissue formation and infiltration of numerous inflammatory cells for 21 days. Moreover, the re-epithelialization was not initiated until 21 DPI. Micrographs of sections in the PC group showed ulcerated surfaces on the 7th day. At the early stage of the healing processes (7 days), the wounds in this group displayed evident inflammatory cell infiltration and granulation tissue formation. However, the inflammatory cells and granulation tissue disappeared quickly for 21 days, and new blood vessels began to grow in this group on the 14th day. Finally, the reepithelialization process was almost completed at 21 DPI.

The evaluation of group O was like that of the group NC on the 7th to 14th days with the presence of the granulation tissue formation and infiltration of numerous inflammatory cells. However, the epithelial layer was started to form on the 21th day as shown in Figure 2. The group P showed the greatest resemblance to normal skin, with less hypertrophic scarring, a thin epidermis, and rejuvenation of skin appendages. Moreover, the re-epithelialization process was initiated on the 14th day (Figure 2).

Overall, the P-treated wounds showed the best results when compared to other experimental groups at 7, 14, and 21 DPI.

The analysis of histological features was performed at 7, 14, and 21 DPI (Table 5). As can be seen in Table 5, group P showed similar epitheliogenesis score with the group PC on the 21th day. However, it demonstrated higher score on the 14th day. Comparison of the results obtained from group P with groups NC and O indicated the higher potency of P than others to induce re-epithelialization.

The inflammation phase is essential for initiating the healing process; however, its prolongation is unwanted. The sharp decrease in the number of inflammatory cells for group P (Figure 3) indicated anti-inflammatory activity of the methanol extract compared with groups PC, O, and NC. In group P, the number of inflammatory cells was significantly decreased from day 7 to day 21 (*P* < 0.01). However, the downward trend showed a steeper slope in the positive control (PC) from day 7 to day 21 (*P* < 0.001). Comparison of the number of inflammatory cells on the 21th day in groups P and O depicted significant decrease of inflammation in group P (*P* < 0.001).

In the case of neovascularization (blood vessels/5HPF), groups P and PC showed desirable changes. For group PC, high neovascularization occurred on the 14th day which was significantly higher than day 7 (*P* < 0.001) and it decreased on the 21th day comparing with the 14th day (*P* < 0.001). However, a downward trend was observed for group P from day 7 to 21 (*P* < 0.001). It seems that the increase of neovascularization occurred before day 7 indicating early proliferative phase. On the other hand, groups NC and O showed increased neovascularization on the day 21 which showed delayed proliferative phase or disrupted remodeling stage.

Analysis of histological features also indicated increase of mature collagen type I in groups P and PC. However, increase of collagen density in group P was significantly higher than the corresponding value for group PC on the same days (*P* < 0.01, *P* < 0.001, *P* < 0.001 for days 7, 14, and 21, respectively). However, the changes in groups O and NC were not significant and no definite pattern was seen.

## 4. Discussion

Wound healing based on natural products has attracted lots of attention both in folk and modern medicine because they are rich in phytochemicals possessing potent anti-inflammatory, antioxidant, antibacterial, and astringent properties, which synergistically play a crucial role in the wound healing cascade. Herein, we focused on the ointment formulation of methanol extract of *C. deodara* wood to evaluate its burn wound healing activity through an *in vivo* burn model in different groups including positive control (PC), negative control (NC), ointment blank (O), and plant extract (P) groups within 21 days. The potent healing properties of *C. deodara* seems to be associated with the presence of phenolic compounds especially flavonoids as reported in Table 1. However, the role of tannins in the healing activity of the plant cannot be ignored. The phytochemical studies of *C. deodara* wood have indicated the presence of flavonoids and flavonols. For example, cedeodarin, dihydromyricetin, cedrin, and cedrinoside have been isolated from the plant [18].

The role of phenolic compounds and tannins in the wound healing process has been fully discussed in the literature. Flavonoids play an important role in angiogenesis, collagen deposition, epithelialization, and wound contraction in the proliferative stage [19]. Also, they have shown antioxidant, antiviral, antimicrobial, anti-inflammatory, and antiproliferative activities, which can accelerate wound healing by the reduction of complications of the process [20]. Tannins also have been documented for their potent antibacterial [21, 22] and antioxidant activities [23], which can improve the wound healing process [24]. They not only heal burn wounds, but they also stop infection along with the healing process. Moreover, they are able to construct a layer over the exposed injury, protecting the tissue from infection [25].

Based on the DPPH radical scavenging assay, the methanol extract of *C. deodara* showed good anti-oxidant activity. As high levels of reactive oxygen species (ROS) complicate the healing process, the healing activity of the plant can be considered from the aspect of anti-oxidant activity [26].

Infections slow down or prevent the healing process. In this respect, antibacterial agents are necessary to stop the bacterial growth as it can lower the wound pH and decrease the oxygen levels. Furthermore, infection can also increase the levels of proinflammatory cytokines, prolonging the inflammatory phase and preventing the proliferative stage from moving on to the remodeling stage [27]. *Staphylococcus* spp. specifically *S. aureus* is a significant cause of infection, strongly in hospitalized patients and fighting against this bacterial strain is important in the healing process [28]. Good anti-bacterial activity of the methanol extract of *C. deodara* against *S. aureus* proves the healing ability.

Good results from phytochemical studies and *in vitro* assays are in good agreement with those obtained from *in vivo* experiment, confirming burn wound healing activity of the methanol extract of *C. deodara* in a topical ointment formulation.

An *in vivo* study within 21 days depicted that the group treated with plant extract (P) showed significantly higher wound closure (%) than the other groups (O, NC, and PC with *P* < 0.001, *P* < 0.001, and *P* < 0.05, respectively).

As reported in Table 5, group P showed much better re-epithelialization than group O and was also comparable with the group PC. It seems that the high content of flavonoids of the studied extract is responsible for the desirable result as the role of flavonoids in enhancing re-epithelialization has been well discussed in the literature [11].

As decreasing the number of inflammatory cells in the wound bed is essential for the progression of the healing process [27], the downward trend for group P from day 7 to day 21 (*P* < 0.01) proves its better healing activity on the 21th day, comparing with groups PC (*P* < 0.05) and O (*P* < 0.001).

Formation of new blood vessels or neovascularization is an essential step in the proliferative phase. In this phase, increasing the number of new blood vessels is vital for providing the necessary nutritional metabolites for the injured tissue. However, this number regresses to the preinjury state moving into the remodeling phase. Failing this process can prolong the proliferative stage and slow down the healing process, creating chronic skin impairments [29, 30]. In this study, treating wounds with the methanol extract of *C. deodara* led to a significant reduction of neovascularization on the 21th day, compared with the 14th day (*P* < 0.001), while the group O demonstrated significant increase in neovascularization on the 21th day, compared with the 14th day (*P* < 0.01), which indicated delay in the proliferative phase or a disruption in the remodeling stage.

It is known that increase of mature type I collagen promotes wound contraction, which was clearly achieved in group P. In this group, a significant early increase of type I collagen density was observed from day 7 to day 14 (*P* < 0.001), depicting significantly higher collagen content on the 14th day, compared with group PC (*P* < 0.001) and O (*P* < 0.001). A significant increase of collagen density was observed from the 14th day to the 21th day in group PC (*P* < 0.05), however, the collagen content of group P on the 21th day was still significantly higher than that of group PC (*P* < 0.001). These results can be attributed to the high flavonoid content since these compounds are known to stimulate biosynthesis of collagen [31].

## 5. Conclusion

The burn wound healing activity of the methanol extract of *C. deodara* wood was studied in a burn wound model using an ointment formulation. It was perceived that the plant can be considered in the development of effective healing agents for treating burns as desirable antioxidant and antibacterial properties were confirmed. Furthermore, the *in vivo* experiment indicated satisfactory results from wound closure percentage, epitheliogenesis score, number of inflammatory cells, neovascularization, and collagen density as the main factors in the wound healing process.

## Figures and Tables

**Figure 1:** *Cedrus deodara* (Roxb. Ex Lamb.) G. Don.

**Figure 2:** Haematoxylin and eosin (H&E) and masson trichrome (MT) stained histopathological sections of the healing incisional wounds. Thick black arrows: crusty scab; white arrows: re-epithelialization; thin black arrows: rejuvenation of skin appendages. Mature collagen type I is shown in blue.

**Figure 3:** The number of inflammatory cells.

**Table 1:** Total phenolic, flavonoid, and tannin contents of methanol extract of *C. deodara*.

Total phenolic content	399.95 ± 19.59 *μ*g GAE^1^/mg dry extract
Total flavonoid content	407.27 ± 5.03 *μ*g CAE^2^/mg dry extract
Total tannin content	9.02 ± 0.17 *μ*g TAE^3^/mg dry extract

^1^GAE = gallic acid equivalent; ^2^CAE = catechin equivalent; ^3^TAE = tannic acid equivalent.

**Table 2:** Antimicrobial activity of methanol extract of *C. deodara* against *Staphylococcus aureus* and *Pseudomonas aeruginosa*.

Sample	MIC (*μ*g/mL)	
	*S. aureus*	*P. aeruginosa*
Extract	625	>2500
Ciprofloxacin	0.78	0.04

**Table 3:** Wound healing activity of the methanol extract of *C. deodara* based on wound surface area^a^.

Area (cm^2^)^b^	P	O	NC	PC
Day 0	3.13 ± 0.06	3.13 ± 0.07	3.14 ± 0.06	3.12 ± 0.06
Day 1^c^	9.97 ± 0.36	10.12 ± 0.18	9.70 ± 0.37	9.73 ± 0.37
Day 7	6.56 ± 0.73	8.08 ± 0.66	7.46 ± 0.74	7.03 ± 1.53
Day 14	1.30 ± 0.39	2.22 ± 0.27	2.59 ± 0.28	1.88 ± 0.29
Day 21	0.67 ± 0.25	1.99 ± 0.23	2.11 ± 0.06	1.14 ± 0.25

^a^Healing activity was investigated using a burn wound model: O = group treated with ointment base with no extract, P = group treated with topical ointment containing extract, NC = group treated with nothing and only dressed in sterile gauze, and PC = positive control. ^b^Reported as mean ± SD. ^c^Post wound expansion.

**Table 4:** Wound healing activity of the methanol extract of *C. deodara* based on wound contraction^a^.

Wound contraction (%)^b^	Day 7	Day 14	Day 21
P	33.6 ± 8.9^ns^	87.1 ± 3.9^*∗*^	93.4 ± 2.4^*∗*^
O	20.1 ± 7.4^ns^	77.9 ± 2.8^ns^	80.2 ± 2.3^*∗∗*^
NC	23.1 ± 7.4^ns^	73.04 ± 2.5^*∗∗*^	78.15 ± 0.4^*∗∗∗*^
PC	27.6 ± 16.4	80.71 ± 2.4	88.35 ± 2.0

^a^Healing activity was investigated using a burn wound model: O = group treated with ointment base with no extract, P = group treated with topical ointment containing extract, NC = group treated with nothing and only dressed in sterile gauze, and PC = positive control. ^b^Reported as mean ± SD. Mean values within each group were compared with PC as the positive control: ns = not significant, ^*∗*^*P* < 0.05, ^*∗∗*^*P* < 0.01, and ^*∗∗∗*^*P* < 0.001.

**Table 5:** Histological features of burn wound healing with different experimental groups.

Groups	Epitheliogenesis score (*n* = 5)	Number of inflammatory cells (×10^3^)^a^	Neovascularization (blood vessels/5HPF)^a,b^	Collagen density (%)^a,b^
PC	0 (7 d)	128.0 ± 5.6 (7 d)	5.2 ± 0.8 (7 d)	29.4 ± 3.8 (7 d)
	1 (14 d)	74.0 ± 9.4 (14 d)	35.2 ± 7.3 (14 d)	39.8 ± 3.7 (14 d)
	4 (21 d)	27.4 ± 4.2 (21 d)	9.0 ± 2.0 (21 d)	50.6 ± 8.79 (21 d)

NC	0 (7 d)	138.6 ± 8.5^ns^ (7 d)	15.2 ± 3.0^*∗∗∗*^ (7 d)	34.4 ± 5.9^ns^ (7 d)
	0 (14 d)	116.2 ± 5.4^*∗∗∗*^ (14 d)	12.2 ± 3.2^*∗∗∗*^ (14 d)	30.6 ± 6.2^ns^ (14 d)
	1 (21 d)	64.8 ± 6.5^*∗∗∗*^ (21 d)	28.0 ± 4.8^ns^ (21 d)	31.2 ± 4.7^*∗∗*^ (21 d)

O	0 (7 d)	115.0 ± 10.5^ns^ (7 d)	8.6 ± 1.8^ns^ (7 d)	39.4 ± 4.8^ns^ (7 d)
	1 (14 d)	100.2 ± 12.2^*∗∗*^ (14 d)	7.2 ± 2.4^*∗∗∗*^ (14 d)	44.0 ± 10.9^ns^ (14 d)
	3 (21 d)	62.2 ± 6.6^*∗∗∗*^ (21 d)	18.6 ± 5.4^ns^ (21 d)	40.8 ± 7.7^ns^ (21 d)

P	0 (7 d)	113.0 ± 14.7^ns^ (7 d)	17.2 ± 2.9^*∗∗∗*^ (7 d)	45.0 ± 7.6^*∗∗*^ (7 d)
	2 (14 d)	87.8 ± 8.8^ns^ (14 d)	14.0 ± 2.7^*∗∗∗*^ (14 d)	74.0 ± 9.4^*∗∗∗*^ (14 d)
	4 (21 d)	17.8 ± 2.6^*∗*^ (21 d)	4.6 ± 1.7^ns^ (21 d)	74.2 ± 5.4^*∗∗∗*^ (21 d)

^a^Mean values within each group were compared with PC as the positive control: ns = not significant; ^*∗*^*P* < 0.05, ^*∗∗*^*P* < 0.01, and ^*∗∗∗*^*P* < 0.001. ^b^Reported as mean ± SD.

## Data Availability

The original datasets supporting the findings of the present study can be obtained from the corresponding author upon reasonable request.
